# Development of a standardized laparoscopic caecum resection model to simulate laparoscopic appendectomy in rats

**DOI:** 10.1186/2047-783X-19-33

**Published:** 2014-06-17

**Authors:** Philipp Lingohr, Jonas Dohmen, Hanno Matthaei, Timo Schwandt, Gun-Soo Hong, Nils Konieczny, Edwin Bölke, Sven Wehner, Jörg C Kalff

**Affiliations:** 1 Department of General, Visceral, Thoracic and Vascular Surgery, University of Bonn, Sigmund-Freud-Strasse 25, 53127 Bonn, Germany; 2 Department of Radiotherapy and Radiation Oncology, University of Düsseldorf, Moorenstrasse 5, 40225 Düsseldorf, Germany

**Keywords:** Laparoscopy, Caecum resection, Rats, Appendectomy, Stump closure, Laparoscopic procedures

## Abstract

**Background:**

Laparoscopic appendectomy (LA) has become one of the most common surgical procedures to date. To improve and standardize this technique further, cost-effective and reliable animal models are needed.

**Methods:**

In a pilot study, 30 Wistar rats underwent laparoscopic caecum resection (as rats do not have an appendix vermiformis), to optimize the instrumental and surgical parameters. A subsequent test study was performed in another 30 rats to compare three different techniques for caecum resection and bowel closure.

**Results:**

Bipolar coagulation led to an insufficiency of caecal stump closure in all operated rats (Group 1, *n* = 10). Endoloop ligation followed by bipolar coagulation and resection (Group 2, *n* = 10) or resection with a LigaSure™ device (Group 3, *n* = 10) resulted in sufficient caecal stump closure.

**Conclusions:**

We developed a LA model enabling us to compare three different caecum resection techniques in rats. In conclusion, only endoloop closure followed by bipolar coagulation proved to be a secure and cost-effective surgical approach.

## Background

Appendicitis remains the most frequent intra-abdominal emergency in humans with approximately 250,000 appendectomies performed in the US every year [1]. Over the past decades, a switch from conventional appendectomy (CA) to laparoscopic appendectomy (LA) has taken place in a majority of modern hospitals around the world [2]. The prevailing advantages of the laparoscopic approach are faster postoperative recovery, a cosmetically more favourable result, shorter hospital stay, reduced postoperative pain, and the ability to inspect the entire abdomen during laparoscopy [3,4]. Nonetheless, primary CA should still be considered in selected patients with contraindications for laparoscopy, such as severe cardiopulmonary disease, or pregnant women, especially in the third trimester.

Despite a high and still growing experience with LA in most modern hospitals, there is still a possibility of significant clinical problems due to this procedure. One of the most feared complications is postoperative insufficiency of the appendiceal stump. This clinical condition leaves the patient at high risk of severe morbidity or even mortality. Given that appendicitis affects mostly younger individuals, complications associated with appendiceal stump insufficiency (e.g. peritonitis with long-term ICU stay, peritoneal adhesions followed by mechanical ileus, incisional hernia, short bowel syndrome after intestinal resections, etc.) may have a large impact on the quality of life of patients for a long period of time and sometimes for the rest of their lives. For this reason, a 100% safe resection and stump closure technique is the foremost goal for every surgeon performing LA.

The first LA was performed by Professor Kurt Semm and colleagues at University of Kiel in 1980 [5]. Since then there has been a massive improvement in both surgical technique and medical products used, minimizing the operative risk. Still, this constant improvement of LA is a work in progress. With respect to the large and still increasing number of LAs performed every year, animal models are expected to be an effective tool for further optimizing this surgical intervention and providing an indispensable source for further analyses regarding cellular and molecular differences (i.e. immune responses, wound healing, vascular perfusion, etc.) between conventional (CS) and laparoscopic surgery (LS).

In our study, we followed this idea and also the hypothesis that a rat model might be ideal for LA research for several reasons. Firstly, it meets the need for a reproducible way to study surgeries in mammals. Secondly, the associated costs can likely be kept at a tolerable level unlike models with larger animals. Thirdly, in general, there are anatomical benefits; although rats do not actually have an *appendix vermiformis* they have a proportionally large caecum, technically facilitating a simulated appendectomy.

Indeed, the idea of using rats to simulate an appendectomy is not new. Several recent studies investigated open caecum resections in rats for this purpose [6-10], some of which examined laparoscopic techniques [11-15]. However, the data available on laparoscopic caecum resection in rats is scarce; small cohorts of animals have been used and incomplete procedural descriptions have been presented by some authors [16-24]. Furthermore, a majority of published operations must essentially be classified as hybrid interventions rather than pure LS [16-22,24]. Polat *et al*. performed actual laparoscopic caecum resections in rats using two endoloops and intracorporeal dissection [23]. Unfortunately, the authors did not describe their operative procedure in sufficient detail for straightforward reproducibility.

Therefore, we sought to establish a reliable and reproducible animal model for implementing laparoscopic partial caecum resection to simulate LA and spent particular attention on an easy-to-perform, reliable, realistic and cost-effective approach to facilitate future research on LA as a commonly performed operation worldwide.

## Methods

### Animals

The present study was approved by the Institutional Review Board as well as by the federal animal research committee (LANUV Nordrhein-Westfalen, Recklinghausen, Germany). For the pilot study we included 30 Wistar Han IGS rats (7 female and 23 male animals) with a median body weight of 439.5 g (range: 170 to 560 g) provided by Charles River WIGA Deutschland GmbH (Bad Königshofen, Germany). In the second part of our project, the actual test study, we operated on another 30 Wistar Han IGS rats (15 male and 15 female animals) with a median body weight of 309.5 g (range: 216 to 416 g). All rats were kept under pathogen-free and standardized conditions (temperature ranging from 20°C to 24°C with 12 hours of light and 12 hours of darkness). We provided free access to food through a standard laboratory diet and water supply *ad libitum* prior to the operation.

### Surgical equipment

All operations were performed under strictly sterile conditions by one experienced laparoscopic visceral surgeon (PL) at the animal operation workplace, House of Experimental Therapy, University of Bonn, Germany. For this purpose, a work station (Figure 1) was designed consisting of a Tele Pack, an Electronic Endoflator® and an Autocon® II 200 (Karl Storz GmbH & Co KG, Tuttlingen, Germany), as well as a warming plate and equipment for anaesthesia. Furthermore, 2- to 5-mm laparoscopic instruments were used (Karl Storz GmbH & Co KG). A LigaSure™ generator, 5-mm LigaSure™ devices and suture material were used within the test study (not shown in the picture, Covidien Deutschland GmbH, Neustadt/Donau, Germany).

**Figure 1:** **Animal operation workplace. (A)** Tele Pack. **(B)** Electronic Endoflator®. **(C)** Autocon® II 200 (Karl Storz GmbH & Co KG , Tuttlingen, Germany). **(D)** Warming plate. **(E)** Equipment for anaesthesia. **(F)** 2- to 5-mm laparoscopic instruments (Karl Storz GmbH & Co KG).

### Laparoscopic surgery performed within pilot study

For the first 30 operations within the pilot study, we sought to test the feasibility of our laparoscopy model. Different techniques and equipment were used to identify the ideal approach for the subsequent experiments described later. These primary operations were initially performed by one surgeon using a camera holder (University of Dundee, Dundee, UK). Due to discomfort, we changed to a two-person procedure for the following 30 procedures in the test study.

The operations were initiated through application of subcutaneous buprenorphine (Temgesic®, Reckitt Benckiser (Deutschland) GmbH, Mannheim, Germany) (0.03 to 0.05 mg/kg) and narcosis was then continued under an isoflurane (Forene®, Abbott GmbH & Co KG, Wiesbaden, Germany) mask. At first, the rats were fixated in front of the mask using a rodent restraint bag and later placed in a dorsal position (Figure 2). The flow of isoflurane (Forene®, Abbott GmbH & Co KG, Wiesbaden, Germany) was started at 3 vol% followed by a reduction to 1.5 vol% with an initial flow of 5 l/min and an additional reduction after 2 min to 2 l/min for the remaining operation. The entire abdomen was shaved and disinfected thoroughly in triplicate using Povidone-iodine. The capnoperitoneum (5 to 7 mmHg using CO_2_) was established using a Veress needle 1 cm subxiphoidally, which was subsequently replaced by a 3-mm trocar. The laparoscope was inserted and an initial four-quadrant laparoscopic inspection was performed. Under videoscopic observation, an additional 2-mm trocar was carefully placed in the left lower abdomen and a 3-mm trocar in the right lower abdomen. All trocars were fixed with a Polysorb™ 3–0 stay-suture (Covidien Deutschland GmbH).

**Figure 2:** **Optimized operative set-up developed during the pilot study.** The rat is in a dorsal position, tail up and head down. Maximum surgical comfort was achieved using a 2.7-mm 30° Hopkins® optic (Karl Storz GmbH & Co KG) in combination with 2- and 3-mm endoscopic instruments (Karl Storz GmbH & Co KG). The photograph shows three trocars: **(A)** 3-mm camera and insufflation trocar, **(B)** 2-mm working trocar and **(C)** 3-mm working trocar.

### Laparoscopic surgery performed within test study

For the second part of our study, we tested three different surgical methods. For Group 1 (ten rats, five female, five male), we used a 3-mm Take-apart® Manhes Bipolar Coagulation Forceps (Karl Storz GmbH & Co KG) for caecum coagulation with 70 mA applied three times for 10 sec in an overlapping manner. For Group 2 (ten rats, five female, five male), a modified Surgitie™ 2–0 (Covidien Deutschland GmbH) was placed at the proximal caecum and the distal part was coagulated (Figure 3). For Group 3 (ten rats, five female, five male), we used a 5-mm LigaSure™ device (Covidien Deutschland GmbH) to close the basis of the appendiceal stump by coagulating twice. Afterwards, the specimens (Figure 4) were resected in all groups in the same manner using 3-mm endo-scissors and extracted through the incision in the right lower abdomen. For this purpose, the incision was slightly dilated from an initial 3 mm to approximately 5 mm. The intraoperative situs, especially the stump, was then thoroughly inspected by laparoscopy to ensure sufficient closure as well as for haemostasis. After removal of the capnoperitoneum, all trocars were removed under vision and the incisions closed in a two-layer manner with interrupted sutures. For the abdominal wall, we used Polysorb™ 3–0 and for the skin we used Monosof™ 4–0 sutures (Covidien Deutschland GmbH).

**Figure 3:** **Example of a laparoscopic caecum resection in an animal from Group 2.** Initially the caecum and the terminal ileum were inspected. **(A)** Avascular plane between both structures (white star). **(B)** The caecum was decompressed using an atraumatic 3-mm grasper (white cross) while it was being held with another 2-mm grasper (white star). **(C)** An endoloop device (white star) was placed proximal to the intended resection site. **(D)** Coagulation of the caecum to prevent any contamination (white star). **(E)** Resection of the caecum (white star) using 3-mm scissors. **(F)** Ligated and coagulated stump (white star), which was inspected to ensure there was sufficient closure and haemostasis.

**Figure 4:** Resected and extracted specimen.

### Postoperative analysis of stump closure integrity

After 60 min, we performed another laparoscopic inspection to check there was sufficient stump closure. Furthermore, a laparoscopic abdominal lavage with 50 ml phosphate-buffered saline (PBS) was performed followed by a final laparotomy. While the rats were still under narcosis, we removed the sutures closing the subxiphoidal and the left lower abdominal trocar sites. This was followed by inserting 50 ml PBS, irrigating the abdominal cavity for 90 s and eventually aspirating the liquid for later microbial analysis. Finally, we performed a median laparotomy followed by a visual check of the stump to examine the sufficiency of the resection site macroscopically. The rats were eventually sacrificed under sufficient general anaesthesia by exsanguination. Aliquots of 200 μl of the harvested irrigation fluid specimens were stored and used for microbiological analysis on McConkey agar plates designed to grow the gram-negative bacteria typically found in faeces. A stool suspension served as a positive control. The plates were then incubated for 48 h under 37.0°C and analysed for bacterial growth after another 12 and 48 h.

### Long-term follow-up

For the long-term follow-up, we took ten additional rats, performed the same operation as in Group 2 and kept them under the standardized conditions described above. On days 3 and 5, we took five rats and performed the above procedure to check stump closure. Afterwards the animals were sacrificed under sufficient general anaesthesia by exsanguination.

### Statistics

Statistical analyses were performed using GraphPad Prism® 4 (GraphPad Software, Inc, San Diego, CA). Comparisons between groups were carried out using analysis of variance (ANOVA) and a *post hoc t*-test. *P* < 0.05 was considered as statistically significant.

## Results and discussion

We started our experiments by testing different surgical instruments (ranging from 2 to 5 mm), different endoscopic cameras (ranging from 2.7 to 5 mm) and different operation settings for the laparoscopic procedures in rats. The use of 5-mm instruments turned out to be uncomfortable since the instruments were rather long and the required trocars were large and heavy. Slight movements of the instruments easily led to a dislocation of the trocars even when they were fixed with stay sutures and the barycentre was not on the same level as the abdominal wall. Also the graspers and scissors were too large for them to be comfortably handled intracorporeally. The operation was difficult to perform and appeared to be unsafe. The 2- and 3-mm endoscopic instruments were shorter, making them easier to handle intracorporeally and therefore they better fitted our needs while simultaneously keeping the procedures safe. One drawback we experienced were difficulties cutting the endoloop or caecum using the 2-mm endo-scissors. This problem was solved when we changed to 3-mm scissors. The cameras tested ranged in size from 5 mm, which provided a very good view but also a large access trauma, to 2 mm, providing a very poor view but less than half of the access trauma. An optimal compromise between both was provided by a 2.7-mm camera.

Finally, we were able to perform safely complete intracorporeally laparoscopic caecum resections. These were most effectively achieved using a 2.7-mm 30° Hopkins® optic (Karl Storz GmbH & Co KG) in combination with 2- and 3-mm endoscopic instruments (Karl Storz GmbH & Co KG) and a 5-mm LigaSure™ device (Covidien Deutschland GmbH).

### Wistar Han IGS rats in study Groups 1 to 3

Thirty Wistar Han IGS rats were divided into three groups of ten animals each (five female and five male rats per group). The ages and weights did not significantly differ among the groups (Table 1). On each working day, one animal from each group (Groups 1 to 3) was operated on to prevent learning-curve effects.

**Table 1:** Parameters for groups 1 to 3 in the test study

**Group (*N *= 10 each)**	**Resection and closure technique**	**Median operation time (min)**	**Maximum length of resected specimen (cm)**	**Sufficient stump closure**	**Microbiological peritoneal test after appendectomy positive growth**
1	Bipolar	34 (range: 21 to 45)	2.45 (range: 1.5 to 3)	0	10/10
2	EL + BP	39.5 (range: 35 to 48)	2.80 (range: 1.8 to 4)	10	0/10
3	LigaSure™ (Covidien)	21.8 (range: 15 to 31)	2.25 (range: 1.5 to 2.7)	10	0/10

ANOVA analysis showed a statistical significance in the median operation time with *P* = 0.0001. There were no statistically significant differences in the maximum lengths of the resected specimens (*P* = 0.0863).

EL + BP: Endoloop combined with bipolar coagulation.

### Operation time and surgical trauma

The median operation times differed among the three groups. The longest operation time was for Group 2 (median: 39.5 min; range: 35 to 48 min) while the shortest operations were performed in Group 3 (median: 21 min; range: 15 to 31 min). ANOVA showed a significant difference in the median operation time with *P* = 0.0001. The *post hoc t*-test revealed a significant difference in the median operation time between Groups 1 and 2 (*P* = 0.0186), Groups 1 and 3 (*P* = 0.0024) and Groups 2 and 3 (*P* < 0.0001). The size of the caecum specimens resected did not differ significantly among the three series (*P* = 0.0863), showing that size variations did not bias the different findings among the groups.

For Group 1, five of the ten stumps were insufficient intraoperatively, resulting in stool release into the abdominal cavity. The relaparoscopy identified stump insufficiency for each of the five remaining rats, as demonstrated by microbiological analysis. For Group 2, intraoperatively as well as during relaparoscopy, no stool was detectable in the abdominal cavity and the microbiological analysis showed the complete absence of bacterial growth on McConkey agar plates. The results for all ten operations were satisfactory. For Group 3, intraoperatively, there was no indication of leakage or damage, and during relaparoscopy the stump closure was sufficient and no stool translocation was macroscopically observed. The latter was confirmed by microbiological analysis.

In a long-term follow-up group (data not shown), there was no macroscopic or microbiological evidence for contamination or leakage of the stump closure. These results indicate that the stump closure technique described in Group 2 was also sufficient after the critical postoperative time of 5 days.

LS is becoming more and more popular and is available in general and visceral surgery departments around the world. There are striking advantages over open surgery, such as faster recovery, less operative trauma and better cosmetic results. However, evidence is missing for whether the surgical trauma of LS leads to differences within the cellular and molecular responses, i.e. the innate immune response or wound healing. To address this question, appropriate animals model are needed. Unfortunately, LS models are rare and inhomogeneous and often of insufficient description. In the present study, we evaluated three different techniques for LA. We have provided detailed instructions and recommendations that are helpful for addressing further LS approaches within animal studies.

An initial literature search identified several studies that provided valuable information for the present research project [11-24]. It can be assumed that a standard laparoscopic procedure was not used for these studies. Most used a hybrid operation, meaning that the investigators resected the caecum extracorporeally, instead of performing complete intracorporeal laparoscopic resections. Only in the study by Polat *et al*. was it identified that an entire laparoscopic caecum resection was performed using two endoloops [23]. Additionally, most studies do not list all operation parameters in detail (such as the way stumps are disinfected, the kinds of trocar or incision that were used and to what extent they enlarged the incision to exteriorize the resectate) (Table 2).

**Table 2:** Studies reporting on laparoscopic caecum resections in rats

**Publication**	**Size of the animal**	**Anaesthesia**	**Pneumoperitoneum**	**Access**	**Angiocatheter**	**Laparoscope**	**Instrument diameter**	**Incision enlargement**	**Type of resection**	**Type of closure**
Allendorf *et al*. 1996 [16]	150 g	Ketamine	4 to 6 mmHg CO_2_	3 ports	Yes (25 gauge)	4 mm	2 × 2 mm	4 mm	Extracorporeal	Ligature
Allendorf *et al*. 1997 [17]	150 g	Ketamine	4 to 6 mmHg CO_2_	3 ports	Yes (25 gauge)	4 mm	2 × 2 mm	4 to 5 mm	Extracorporeal	Ligature
Le Moine *et al*. 1998 [18]	unknown	Ketamine	12 mmHg CO_2_	3 trocars	No	unknown	unknown	unknown	Extracorporeal	Ligature
Jacobi *et al*. 2001 [19]	unknown	Barbiturate	8 mmHg CO_2_/Helium	3 trocars	No	5 mm (uncertain)	unknown	1 cm	Extracorporeal	Suture
Opitz *et al*. 2003 [20]	250 to 300 g	Barbiturate	8 mmHg CO_2_	1 trocar, 2 ports	No	3.5 mm	2 × 3.5 mm	unknown	Extracorporeal	Suture
Lee *et al*. 2003 [21]	unknown	Ketamine	4 mmHg CO_2_	2 incisions	Yes (18 gauge)	5 mm	1 × 2 mm	unknown	Extracorporeal	Ligature
Bobrich *et al*. 2007 [22]	250 to 300 g	Barbiturate	8 mmHg CO_2_	3 trocars	No	3.5 mm (uncertain)	unknown	unknown	Extracorporeal	Suture
Polat *et al*. 2008 [23]	300 to 350 g	Ketamine	4 to 6 mmHg CO_2_	unknown (3 accesses)	Yes (25 gauge)	4 mm	2 × 2 mm	4 mm (uncertain)	Intracorporeal/extracorporeal	Loop suture/ligature
Schmelzer *et al*. 2008 [24]	unknown	Isoflurane	4 mmHg CO_2_	1 trocar, 1 incision	No	3 mm	1 × 2 mm	1 cm	Extracorporeal	Ligature

Furthermore, the technical and procedural approach varied among the published studies. While most investigators used barbiturate [19,20,22] or ketamine [16-18,21,23] for narcosis, we used isoflurane (Forene®, Abbott GmbH & Co KG, Wiesbaden, Germany), which was also used by Schmelzer *et al*. [24]. We found that this narcosis was easy to handle, very reliable and the rats recovered quickly afterwards. Overdoses or even narcosis-related deaths were not observed.

Regarding the capnoperitoneum, several investigators used an angiocatheter (18 or 25 gauge) in a trocarless method to insufflate the peritoneal cavity [16,17,21,23], while others used proper trocars [18-20,22,24]. As the usage of trocars appears to imitate LA more realistically in comparison with modern human laparoscopy, we consequently used trocars within the present study. Trocar usage was comfortable and ensured a constant capnoperitoneum without loss of pressure. Furthermore, different laparoscopes were used in the studies, ranging in size from 3 mm [24] to 5 mm [19,21]. In our opinion, a 2.7-mm laparoscope is the ideal solution since it provides a compromise between the improved view from the 5-mm laparoscope and the lower access trauma of the 2-mm laparoscope. We suppose that the rapid and constant technological progress will give better vision even using small calibre laparoscopes in the future. Additionally, we found that instrument size is a crucial factor in rat LS, which was unfortunately not explicitly listed in a number of previous publications. Three studies used 2-mm forceps and scissors [16,17,23] and another group 3.5-mm forceps and scissors [20], while two other groups performed their operations with 2-mm forceps [21,24]. To extract the specimen, some investigators needed a 4-mm incision [16,17,23] while others required a widening of 1 cm [24]. We compared several instrument sizes and found that 2-mm and 3-mm laparoscopic instruments and trocars were the ideal size for high-precision interventions while keeping the operative trauma at the lowest possible level. Based on the results of this instrument comparison, we strongly recommend usage of a 2.7-mm laparoscope and 2- to 3-mm instruments for LA. Furthermore, the present instrument setting, particularly the choice of appropriate calibres of laparoscopic instruments, appears to be transferable to other experimental laparoscopic animal models.

After establishing an appropriate instrument setting, we compared three different kinds of appendectomy and stump closure techniques. The only group for which stump insufficiencies were observed was Group 1, in which we used bipolar coagulation. Of note, all animals in Group 1 demonstrated stump insufficiencies. Conflictingly, Aslan *et al*. [11] had sufficient stump closures using a bipolar coagulation device in a previous rat study. Although the bipolar coagulation devices differed between the studies, Take-apart® Manhes Bipolar Coagulation Forceps (Karl Storz GmbH & Co KG) versus Power Blade™ (Lina Tripol 5, Denmark) [11], our results demonstrate severe failure in sufficient stump closure when using only bipolar coagulation for bowel resection surgery. This is confirmed by bursting pressure experiments in the study by Aslan *et al*., which demonstrated a significant decrease in bursting pressure to levels as low as 11 cm H_2_O for bipolar-coagulated stumps. In contrast, for Groups 2 and 3, all stumps were sufficiently closed and no peritoneal bacterial contamination was detected, indicating that the stumps were effectively sealed. The fastest and most comfortable operations were performed with the 5-mm Ligasure™ device for Group 3, although this is also the most expensive technique. Since for Group 2, all stump closures were sufficient and the procedure is the closest to reality, as it is comparable to the one most often used in children, we recommend the use of an endoloop plus bipolar coagulation. This procedure can be performed easily and appears to be safe and cost-effective, at least for research purposes.

One should note that our present study did not include long-time observation of anastomotic stump closure in all groups. We only pursued 3- and 5-day follow-up inspections for Group 2 as this procedure turned out to be the most reliable technique, particularly in terms of safety, simulating reality and cost-effectiveness. Additionally, we are currently not able to adapt the most frequently used appendiceal stump closure techniques for LA for adult humans, because the linear stapler tools used have diameters that are too large (10 mm) and would lead to inappropriate large access traumas in a rat model.

Appendectomy models have historically been useful in a variety of research fields. In CA models, for example, electrosurgical devices (bipolar cautery [11,14], LigaSure Precise [12,14]), endoclips [12-14], endoloops [13,23] and staplers [13,15] have been compared, and all investigated methods have been shown to be feasible, safe and leakproof. While some of the LA rat models also investigated caecum resection and closure techniques, other groups focused on topics such as postoperative immune function [16,17,21,24], risk of neoplastic port site metastasis after LS [18,23], influence of taurolidine/heparin on local tumour growth after laparoscopy [20,22] and postoperative adhesion formation [19]. With our standardized model, we hope to facilitate such research in the future to improve LS.

In the present study, we present evidence to show that endoloop ligation combined with bipolar coagulation is the most appropriate and easy-to-learn model for LA and we hope that this technique will be helpful and further improve research in the field of LA.

## Conclusions

In conclusion, we present an LA model with rats aiming for a surgical approach that is straightforward to reproduce, safe to perform and cost-effective and which is close to the reality of human appendectomies. This work includes a comparative test of instruments, which identified the optimal calibre and length of laparoscopic equipment for LA procedures. We feel that our standardized LA rat model will be beneficial for future appendectomy and LS research.

## Abbreviations

ANOVA: analysis of variance; CA: conventional appendectomy; CS: conventional surgery; LA: laparoscopic appendectomy; LS: laparoscopic surgery; PBS: phosphate-buffered saline.

## Competing interests

This project was supported by the German Research Foundation (Deutsche Forschungsgemeinschaft) and the Bonfor Research Commission. JD is supported by a Bonfor doctoral thesis scholarship. All instruments and operative equipment were kindly provided by Karl Storz GmbH & Co KG (Tuttlingen, Germany) and Covidien Deutschland GmbH (Neustadt/Donau, Germany). There are no competing financial interests and all authors declare there are no competing interests. We presented this model at the 21st International Congress of the European Association for Endoscopic Surgery (EAES) in Vienna, Austria, and won the poster prize.

## Authors’ contributions

PL planned and developed the project, performed the operations, evaluated the results and wrote the manuscript. JD supported the lab work, assisted in the operations and gave support in evaluating the results and writing the manuscript. HM corrected and wrote parts of the manuscript, and gave advice and support in performing the laboratory procedures. GH, TS and NK gave advice and support in performing the laboratory procedures. EB, SW and JCK helped in conceptual project development and writing the manuscript. All authors read and approved the final manuscript.
